The article "Potential Molecular Mechanism of Guishen Huoxue Decoction against Intrauterine Adhesion Based on Network Pharmacology" was retracted in 2023. Reasons: signs of a paper mill; compromised peer review; unreliable results or conclusions.

# Potential Molecular Mechanism of Guishen Huoxue Decoction against Intrauterine Adhesion Based on Network Pharmacology

**DOI:** 10.1155/2022/4049147

**Published:** 2022-09-23

**Authors:** Wenyan Zhang, Yuan Yuan, Guangrong Huang, Jing Xiao

**Affiliations:** ^1^Department of Gynaecology, The Second Clinical College of Guangzhou University of Chinese Medicine, Guangzhou, China; ^2^Department of Gynaecology, Shenzhen Bao'an Chinese Medicine Hospital, Guangzhou University of Chinese Medicine, Shenzhen, China; ^3^Department of Gynaecology, The Second Affiliated Hospital of Guangzhou University of Chinese Medicine, Guangzhou, China

## Abstract

**Objective:**

Intrauterine adhesion (IUA) represents an endometrial repair disorder that is associated with menstrual disorders, recurrent pregnancy loss, and infertility. This study aimed to explore the underlying biological mechanisms of Guishen Huoxue decoction for the treatment of IUA based on network pharmacology.

**Methods:**

The selection of active compounds for Guishen Huoxue decoction and prediction of relevant targets were performed by the TCMSP and Swiss Target Prediction databases, respectively. The targets of IUA were obtained by three databases, including Online Mendelian Inheritance in Man (OMIM), DisGeNET, and GeneCards. The drug-disease regulatory network was constructed via Cytoscape software, following the acquisition of common genes of active compounds of drug Guishen Huoxue decoction and disease IUA, which was carried out through Venny software. Protein-protein interaction (PPI) network and function enrichment analyses were performed.

**Results:**

According to the data obtained from TCMSP, a total of 200 potential active compounds of Guishen Huoxue decoction and their related targets (1068) were screened by the Swiss Target Prediction database. 1303 disease targets and 134 common targets were identified. The drug-disease regulatory network showed that 165 active compounds were found to be involved in the treatment of IUA. Among 134 common targets, AKT1, SRC, TP53, VEGFA, and IL-6 were predicted as core genes against IUA. PI3K-Akt, Rap1, Ras, and AGE-RAGE were the main signaling pathways that participated in the treatment of Guishen Huoxue decoction for IUA.

**Conclusion:**

The active compounds of Guishen Huoxue decoction confer therapeutic effects against IUA by regulating fibrosis, inflammation, and oxidative stress through major signaling pathways such as PI3K-Akt and AGE-RAGE.

## 1. Introduction

Intrauterine adhesion (IUA), also known as endometrial fibrosis or Asherman's syndrome, was first proposed by Joseph Asherman in 1948 [1]. IUA is deemed to be the injury of the endometrial basal layer and partial or complete loss of the functional layer due to various reasons, which eventually leads to adhesion of the uterine walls and partial or even complete occlusion of the uterine cavity [2]. With the increase in abortion and intrauterine surgery, the incidence rate of IUA is increasing year by year, reaching as high as 25%–30% [3]. Endometrial trauma caused by surgery, including abdominal and hysteroscopic myomectomy, septectomy, and any other intrauterine surgery, is the leading contribution to the occurrence of IUA [4]. IUA has become a common gynecological disease and is characterized by a series of clinical manifestations such as oligomenorrhea, dysmenorrhea, amenorrhea, recurrent abortion, and infertility, posing serious damage to women's reproductive function [5, 6]. Previous studies have shown that hysteroscopic adhesiolysis was most commonly used for the clinical treatment of IUA, with the placement of antiadhesion biological adhesive products in the intrauterine cavity and location of intrauterine devices for 2 to 3 months, or retention of the sacculus in the intrauterine cavity for 5–7 days and oral therapy of estrogen and progesterone drugs for 3 months after surgery [7, 8]. However, the recurrence rate of IUA after hysteroscopic adhesiolysis reached 62.5% [9], and the success rate of pregnancy remained approximately 22.5%∼33.3% [10, 11]. Therefore, exploring clinical adjuvant therapy for IUA is necessary.

No descriptions of IUA were found in ancient traditional Chinese medical books, but the symptoms of IUA belong to the categories of “hypomenorrhea,” “amenorrhea,” “abdominal pain,” and “infertility” in traditional Chinese drugs. Most studies believed that this disease was caused by operations in the intrauterine, and the operations damaged the uterus and uterine vessels, resulting in kidney deficiency, insufficiency of vital energy and blood, and blockage of blood stasis [12, 13]. Modern pharmacological studies have shown that kidney tonifying herbs improved endometrial blood supply and elevated the embryo quality in the cycle of controlled ovarian hyperstimulation of assisted reproductive technique [14]. Traditional Chinese herbs provide a new clinical method for the treatment of low endometrial receptivity [15]. Bushen Huoxue decoction can favor decidual stromal cell proliferation and show therapeutic potential to manage patients with unexplained recurrent spontaneous abortion, and its effect was realized through the PI3K/AKT pathway [16]. Traditional Chinese drugs referring to blood circulation promotion and blood stasis removal are helpful to improve local microcirculation, reduce inflammatory reactions, and boost the restoration of the endometrium. Guishen Huoxue decoction, as a term for a series of traditional Chinese drug formulas, is similar to Bushen Huoxue decoction [17] and is effective in blood circulation promotion and kidney tonification. However, no direct evidence of Guishen Huoxue decoction in IUA treatment was found.

Network pharmacology is a new discipline used to analyze the network of biological systems and select specific signal nodes to design multitarget drug molecules [18]. This study was aimed at investigating the potential molecular mechanisms of Bushen Huoxue decoction on the treatment of IUA through network pharmacology and providing ideas for further experimental research and the development of new drugs for the treatment of IUA.

## 2. Materials and Methods

### 2.1. Screening of Drug-Related Active Compounds and Potential Targets

The traditional Chinese drug systems pharmacology database and analysis platform (TCMSP) (https://tcmspw.com/tcmsp.php) was performed to obtain the active compounds of Guishen Huoxue decoction, consisting of *Paeonia lactiflora*, *Ligusticum wallichii*, root of red-rooted salvia, *Angelica sinensis*, fruit of Chinese wolfberry, *Astragalus membranaceus*, Spatholobus stem, fruit of glossy privet, Chinese yam, fruit of medicinal cornel, prepared rehmannia root, seed of Chinese dodder. Oral bioavailability (OB) ≥ 30% and drug-like (DL) ≥ 0.18 were considered the screening conditions of the main active compounds, and the potential targets of the screened compounds were identified using the Swiss Target Prediction (https://swisstargetprediction.ch/) database, with a prediction score greater than zero. The UniProt database (https://www.uniprot.org/) was used for converting target information into gene symbols.

### 2.2. Prediction of IUA Targets

Databases including Online Mendelian Inheritance in Man (OMIM) (https://omim.org/), DisGeNET (https://www.disgenet.org/), and GeneCards (https://www.genecards.org/) were carried out to obtain the disease-related targets (only “*Homo sapiens*”) using “Asherman's Syndrome” and “intrauterine adhesion” as the keywords. A gene symbol was obtained with the help of the UniProt database (https://www.uniprot.org/).

### 2.3. Acquisition of Drug-Disease Common Targets and Drug-Targets-Disease Network Construction

The Venny 2.1 software was performed to acquire common targets of active compounds of the drug Guishen Huoxue decoction and disease IUA. Subsequently, the targeting relationship between active compounds of Guishen Huoxue decoction and common targets was presented by the drug-targets-disease network through Cytoscape 3.7.2 software.

### 2.4. Protein-Protein Interaction (PPI) Network Construction and Screening of Core Genes

The PPI network was constructed based on common targets of Guishen Huoxue Decoction and IUA mapping into the STRING database (https://string-db.org/), with the parameter of “*Homo sapiens*” as protein type and “moderate confidence” (>0.400) as the minimum interaction critical value. The PPI network was visualized by importing the TSV-based file to Cytoscape 3.7.2 software, and the visual analysis included a topology analysis, gene cluster analysis, and core gene screening. On the basis of the degree value obtained, the core genes were sorted out.

### 2.5. Gene Ontology (GO) Function and (Kyoto Encyclopedia of Genes and Genomes) KEGG Pathway Enrichment Analysis

The primary biological process and related signal pathways of Guishen Huoxue decoction in the treatment of IUA were explored by functional enrichment analysis. On the basis of R software, Bioconductor software (*p* value < 0.05, *q* value < 0.05) was applied to perform the GO and KEGG analysis of common targets of Guishen Huoxue decoction and IUA. Go enrichment analysis clarified gene function from three aspects: biological process (BP), cellular component (CC), and molecular function (MF). KEGG reflects a particular pathway of diseases with significant gene concentrations.

## 3. Result

### 3.1. Main Active Compounds and Targets of Guishen Huoxue Decoction

As listed in Table 1, with the help of TCMSP and a condition of OB ≥ 30% and DL ≥ 0.18, it was observed that a total of 200 potential active compounds of Guishen Huoxue decoction (*Paeonia lactiflora*, *Ligusticum wallichii*, root of red-rooted salvia, *Angelica sinensis*, fruit of Chinese wolfberry, *Astragalus membranaceus*, Spatholobus stem, fruit of glossy privet, Chinese yam, fruit of medicinal cornel, prepared rehmannia root, seed of Chinese dodder) were found following duplicate removal. A total of 1169 targets related to potential active compounds were screened using the Swiss Target Prediction database.

### 3.2. Identification of IUA Targets

Using “Asherman syndrome” and “intrauterine adhesions” as the searching keywords, the results of three databases, including OMIM, DisGeNET, and GeneCards, indicated that 1303 disease-related records were obtained after duplicate removal.

### 3.3. Drug-Disease Common Targets and Drug-Targets-Disease Network Construction

The Wayne diagram was mapped using 1169 targets associated with potential active compounds of Guishen Huoxue decoction and 934 disease-related IUA targets via Venny 2.1 software. A total of 134 common target genes were shown in the Wayne diagram (Figure 1). The drug-targets-disease network was established through Cytoscape 3.7.2 software, with the use of 200 potential active compounds and 134 common targets obtained from Guishen Huoxue decoction and IUA, and in the absence of those active compounds that do not intersect with these targets (Figure 2). In Figure 2, the symbols in purple color represented drugs. The green color indicated active compounds of Guishen Huoxue decoction, of which 35 active compounds were deleted due to no commonality with the 134 targets expressed in blue color, and the red color represented disease IUA.

### 3.4. PPI Network Construction and Core Genes Selection

The PPI network (Figure 3), containing 134 common genes in Guishen Huoxue decoction and IUA, was constructed through the STRING database, and then the visualization analysis of PPI was carried out via Cytoscape software, with the confidence score not less than (Figure 4). In the PPI network, the size and color of the nodes were associated with degree values, and the edges indicated the interaction. “Network Analyzer” in Cytoscape software was used for topology analysis of the PPI network. The target proteins whose degree values were greater than the average values were selected as the core proteins, and the first 30 proteins, were plotted using R 3.6.1 software (Figure 5). Among the 30 proteins, 5 proteins were predicted to be core proteins which were screened by the “MCODE tool” in Cytoscape software, and the corresponding gene symbols were AKT1, SRC, TP53, VEGFA, and IL-6.

### 3.5. Enrichment Analysis of Drug-Disease Common Targets

The GO enrichment analysis was conducted following the performance of the R language on 134 common genes. Go analysis indicated that the common genes were enriched in 2291 BP terms, mainly including peptidyl-tyrosine phosphorylation, peptidyl-tyrosine modification, and positive regulation of cell adhesion (Figure 6(a)). In terms of CC, the common genes were associated with 69 terms, such as membrane raft, membrane microdomain, and membrane region (Figure 6(b)). The common genes were mostly enriched in 138 MF terms, such as protein tyrosine kinase activity, transmembrane receptor protein tyrosine kinase activity, and phosphatase binding (Figure 6(c)). After KEGG pathway analysis, the first 20 significant enrichment signal pathways were screened and associated with drug-disease common targets (Figure 7).

## 4. Discussion

IUA is mainly characterized by hypomenorrhea or amenorrhea [6]. The purpose of IUA treatment is to control relevant symptoms, promote endometrial repair and regeneration, and reduce the incidence of readhesion as well as complications such as recurrent abortion and secondary infertility. Although hysteroscopic adhesiolysis as the main treatment is able to restore anatomical morphology of the uterine cavity and uterine cavity volume, it is not an ideal intervention for IUA due to poor recovery of menstruation and fertility, especially an extremely high recurrence rate in the presence of various approaches to prevent recurrent adhesion [19, 20]. Hence, exploring effective adjutant approaches following hysteroscopic adhesiolysis contributes to women's health.

In recent years, traditional Chinese drugs have enriched the development of therapy for uterus-related diseases. Ding et al. revealed that as a classic traditional prescription, Bushen Huoxue Huatan decoction improved polycystic ovary syndrome through regulating hormones, reversing insulin resistance, and alleviating inflammation reactions, resulting in fertility improvement [21]. Feng et al. also proved that Bushen Huoxue decoction was effective in the treatment of unexplained recurrent spontaneous abortion via activation of the PI3K/AKT pathway [16]. The traditional Chinese drug Tiaoshen Tongluo, which contained ingredients associated with the alleviation of fibrosis, was confirmed to attenuate endometrial fibrosis in a rat with IUA through TGF-*β*1/Smad Pathway [22]. Similarly to Bushen Huoxue decoction, Guishen Huoxue decoction is a traditional drug formulation, consisting of *Paeonia lactiflora*, *Ligusticum wallichii*, the root of red-rooted salvia, *Angelica sinensis*, fruit of Chinese wolfberry, *Astragalus membranaceus*, Spatholobus stem, fruit of glossy privet, Chinese yam, fruit of medicinal cornel, prepared rehmannia root, seed of Chinese seed of Chinese dodder, improves renal function and promotes blood circulation [23, 24].

In this study, we performed drug-disease regulatory network construction and the PPI network construction to obtain the core genes of Guishen Huoxue decoction for the treatment of IUA, and the core genes were analyzed by GO function enrichment and KEGG pathway enrichment to explore their potential molecular mechanisms. A total of 134 common targets were obtained from Guishen Huoxue decoction and IUA, and five core genes, including AKT1, SRC, TP53, VEGFA, and IL-6, were mainly enriched in PI3K/Akt, Rap1, Ras, and AGE-RAGE signaling pathways. IUA is a fibrotic disease, that is, the serious damage of the endometrial basal layer promotes a large number of fibrocyte proliferations and excessive deposition of extracellular matrix, leading to the partial or complete replacement of endometrial tissue by fibrous tissue [25]. VEGF is the major inducer of angiogenesis in a variety of in vivo models and plays an essential role in numerous physiological and pathological processes, including angiogenesis and immune response [26, 27]. Increased expression of VEGF has been reported to alleviate endometrium injury in a wounded rat uterus [28]. The patients with IUA showed vascular closure in endometrial tissues and had significantly increased VEGF expression after therapy, suggesting angiogenesis in the endometrial tissues may affect the endometrial repair [29]. A series of abnormal inflammatory cells and inflammatory responses in the uterine cavity promote the development of fibrosis. A in vivo experiment described by Ai et al. [30] demonstrated that alleviation of the inflammatory response and epithelial-to-mesenchymal transition process enhanced endometrium regeneration rats. IL-6 is a typical cytokine that maintains homeostasis and contributes to host defense by activating acute phase responses and hematopoietic and immune responses [31]. IL-6 and IL-10 levels were associated with endometrial lesions in equines, which can be considered as inflammatory indexes to evaluate the pathological progress of the equine endometrium [32]. The role of AGE-RAGE signaling has been demonstrated in the progression of various diseases such as diabetes, cardiovascular diseases, neurodegenerative disorders, and cancer [33]. Studies have found that increased levels of AGE and its receptor RAGE are associated with ovarian senescence and induce inflammatory responses [34].

AKT1 plays a key role in cell growth and survival in various diseases. Nie et al. manifested that [35] AKT1 mediated the progression of idiopathic pulmonary fibrosis by inducing macrophages to produce IL-13. PI3K/Akt mediates cell apoptosis, proliferation, and differentiation of bone marrow stem cells and endothelial progenitor cells and was involved in IUA pathogenesis [36]. Rap1 and Ras regulate cell development and participate in the growth and survival of normal and cancer cells[37]. The Rap1 signaling pathway is involved in the cAMP-mediated decidualization of human endometrial stromal cells [38]. The Ras signaling pathway medicates the pathogenesis of RIF induced by endometrial receptivity insufficiency and regulates Talin1 expression (a local adhesion complex protein) in the endometrium. Steroid hormones, including estrogen and progesterone, are involved in mammalian reproduction and regulate the development and function of the uterus by mediating the transcription of specific genes in the uterus [39]. As the largest nonreceptor tyrosine kinases, SRC and SRC family kinases are proto-oncogenes that play vital roles in cell proliferation, invasion and metastasis, angiogenesis, and bone metabolism [40]. Furthermore, SRC family kinases have been identified to be related to the function of steroid responses [41], and SRC activation is critical for decidualization, maintaining remodeling, and differentiation of the estradiol-primed endometrium [42]. It was reported that the TP53 gene, as a tumor suppressor, has mutated in more than 45,000 single cell and germline mutations, accounting for more than 50% of human tumor gene mutations [43], including endometrial cancer [44]. TP53 function loss leads to endometrial hyperplasia and promotes aggressive or metastatic endometrial cancers [45].

In summary, our study based on network pharmacology shows that AKT1, SRC, TP53, VEGFA, and IL-6 in Guishen Huoxue decoction might be potential biomarkers for the treatment of IUA, and Guishen Huoxue decoction regulates fibrosis, inflammatory response, and oxidative stress response through several main signaling pathways including PI3K-Akt, Rap1, Ras, and AGE-RAGE. This study has conducted a preliminary theoretical discussion on the use of Guishen Huoxue decoction in the treatment of IUA. In the future, we need to verify our results through molecular docking analysis of drug-disease targets and active chemical compounds as well as experimental validation in cell and animal models.

## Figures and Tables

**Figure 1:** Screening of common targets existing in Guishen Huoxue decoction and disease IUA. The circle in purple means targets of active compounds in Guishen Huoxue decoction, and the circle in yellow represents targets of disease in IUA.

**Figure 2:** Regulatory networks between Guishen Huoxue decoction and IUA. The symbols in purple color represent drugs. The green color indicates active compounds in the Guishen Huoxue decoction. Common targets are expressed in the blue color. The red color meant disease IUA.

**Figure 3:** PPI network constructions.

**Figure 4:** PPI network visualization analyses. The nodes represent the targets, and the size and color shades show their degree in the network.

**Figure 5:** Screening of the top 30 genes based on the PPI topology analysis.

**Figure 6:** GO functional enrichment analyses of common genes. Significant enrichment of common genes in MF (molecular function) category (a), CC (cellular component) category (b), and BP (biological process) category (c) (the top 20 GO terms for each category are listed).

**Figure 7:** KEGG pathway enrichment analysis of common genes. The red color indicates a small *p* value and the blue color indicates a large *p* value; the size of the bars represents the degree of enrichment, and larger bars reflect a larger gene ratio.

**Table 1:** Drug-related active compounds and potential targets.

Drug	Numbers of active compounds	Numbers of targets
*Paeonia lactiflora*	13	342
Ligusticum wallichii	7	349
*Salvia miltiorrhiza*	65	716
Chinese angelica	2	43
Fruit of Chinese wolfberry	45	423
*Astragalus membranaceus*	20	429
Spatholobus stem	24	502
Fruit of glossy privet	13	231
Chinese yam	16	334
Fruit of medicinal cornel	20	358
Prepared rehmannia root	2	44
Seed of Chinese dodder	11	279

## Data Availability

The data used to support the findings of this study are included within the article.
